The article "A Computationally Virtual Histological Staining Method to Ovarian Cancer Tissue by Deep Generative Adversarial Networks" was published in 2021. Journal: Comput Math Methods Med.

# A Computationally Virtual Histological Staining Method to Ovarian Cancer Tissue by Deep Generative Adversarial Networks

**DOI:** 10.1155/2021/4244157

**Published:** 2021-07-01

**Authors:** Xiangyu Meng, Xin Li, Xun Wang

**Affiliations:** ^1^College of Computer Science and Technology, China University of Petroleum, Qingdao, 266580 Shandong, China; ^2^College of Computer and Information Science, Inner Mongolia Agricultural University, Huhhot, 010018 Inner Mongolia, China; ^3^Department of Gynecology 2, Renmin Hospital of Wuhan University, Wuhan, 430060 Hubei, China; ^4^China High Performance Computer Research Center, Institute of Computer Technology, Chinese Academy of Science, Beijing, 100190 Beijing, China

## Abstract

Histological analysis to tissue samples is elemental for diagnosing the risk and severity of ovarian cancer. The commonly used Hematoxylin and Eosin (H&E) staining method involves complex steps and strict requirements, which would seriously impact the research of histological analysis of the ovarian cancer. Virtual histological staining by the Generative Adversarial Network (GAN) provides a feasible way for these problems, yet it is still a challenge of using deep learning technology since the amounts of data available are quite limited for training. Based on the idea of GAN, we propose a weakly supervised learning method to generate autofluorescence images of unstained ovarian tissue sections corresponding to H&E staining sections of ovarian tissue. Using the above method, we constructed the supervision conditions for the virtual staining process, which makes the image quality synthesized in the subsequent virtual staining stage more perfect. Through the doctors' evaluation of our results, the accuracy of ovarian cancer unstained fluorescence image generated by our method reached 93%. At the same time, we evaluated the image quality of the generated images, where the FID reached 175.969, the IS score reached 1.311, and the MS reached 0.717. Based on the image-to-image translation method, we use the data set constructed in the previous step to implement a virtual staining method that is accurate to tissue cells. The accuracy of staining through the doctor's assessment reached 97%. At the same time, the accuracy of visual evaluation based on deep learning reached 95%.

## 1. Introduction

Computer-aided medical diagnosis is a hot topic nowadays. In recent years, researchers devoted to the issue in this direction and achieved excellent research outcomes. Some studies [1–5] established spiking neural networks to simulate biological metabolic processes, infer the final physiological calculation results, and obtain the final diagnosis solution. Some studies [6–10] rely on the idea of deep learning to build a deep neural network model to complete the diagnosis of patients based on the characteristics of various medical data. The above methods have achieved extraordinary accuracy and efficient treatment for specific medical domain. However, few studies have focused on the preparation and labeling of medical data. At present, traditional medical data preprocessing methods can no longer meet the needs of intelligent diagnosis with large data volumes.

The ovarian cancer is a global problem, is typically diagnosed at a late stage, and has no effective screening strategy [11]. Microscopic imaging of tissue samples is the basis for subsequent diagnosis and prognosis of cancer. H&E staining and labeling of tissue samples can better help locate suitable cancer tissues and perform subsequent analysis, diagnosis, and prognosis. Therefore, strict control of tissue section staining standards will significantly enhance the final diagnosis and prognosis results. However, the traditional histopathological section staining process involves many standard operating steps, and each technician must strictly adhere to these gold standards. These methods are often time-consuming and laborious and often have higher requirements. The histological tissue appearance may assume different color intensities depending on the staining process, operator ability, and scanner specifications [12]. The above problems will seriously harm the analysis of the disease pathology of the tissue and the events of the disease prognosis. Many coping strategies have been established to improve the success rate and quality of tissue staining in clinical trials. Massimo et al. [12] presented a novel fully automated stain separation and normalization approaches for Hematoxylin and Eosin stained histological slides to improve the contrast between histological tissue and background and preserve local structures without changing the color of the lumen and the background. Mario et al. [13] used experiments to clarify Eosin-based fluorescence spectroscopy can be used to directly examine H&E stained tissue slides. Relevant areas can be imaged and spectral analysis done to obtain objective data. The above method does solve the problems of low accuracy and poor effect in traditional staining to a certain extent. However, the first method still cannot avoid the strict and complicated processing steps of the traditional method. Although the second method uses a more novel method of labeling pathological tissues, the use of H&E staining analysis is still the mainstream processing method for pathology research today. The popularization and promotion of this program are still a long process.

We propose to construct a computationally staining and labeling algorithm for H&E staining of the ovarian cancer tissue sections. This method can effectively avoid the complicated steps of H&E staining of traditional ovarian cancer tissue sections and make up for the diagnosis tension caused by the lack of data. Rivenson et al. [14] proposed a virtual staining method for pathological sections based on deep learning. They placed the fresh tissue section on a fluorescence microscope to observe the autofluorescence imaging of the tissue sample and then stained and labeled the sample to obtain the corresponding stained image. After repeating the above work, a huge data set is constructed, and then, a deep learning model is performed to complete the feature learning from unstained samples to stained samples. However, the above method requires a large number of tissue samples from the patient and cannot be effectively implemented under multiple limited conditions. At the same time, the process of data construction still cannot completely get rid of the traditional H&E staining process.

To solve the problems above, we firstly proposed a weakly supervised image generation algorithm based on the CycleGAN model [15], which generate the corresponding unstained image for the stained ovarian sections.  Figure 1(a) shows the overview of this domain translation method. We introduce the domain consistency loss based on the original CycleGAN model, to ensure that the results after the cycle generation are accurately matched to the specific domain. The introduction of input buffers can better magnify the effect of domain consistency loss. We only collected 400 H&E staining images of ovarian cancer and 80 autofluorescence images from other tissues as the experimental data set. From the experimental results, it can be seen that under such extremely inconsistent distribution conditions, the construction of H&E staining images to corresponding unstained images can be completed based on our method. The data set constructed by the above method can provide a good data guarantee for this goal.  Figure 1(b) shows the overview of the virtual staining process. We analyzed whether the state-of-the-art image translation model can be effectively used in this experimental environment, but it is a pity that although these methods have some effects, they cannot meet our requirements for absolute fineness. Therefore, we made improvements on the traditional UNet basic framework [16] and proposed the Parallel Feature Fusion Network (PFFN). At the same time, we introduced a more superior training method to better fit the model to the optimal state. Compared with the traditional image translation method, the quality of the image generated by our improved image translation method is superior.

In this work, we mainly solved two problems. The first is that due to the limited number of pathological tissue samples, we provide a method for constructing a virtual data set composed of autofluorescence imaging of ovarian cancer pathological tissues and corresponding H&E staining imaging. Using our method, limited ovarian tissue images can be augmented with high quality in a short time. Next, based on our augmented data, we propose a virtual staining method. Using this method can swiftly and efficiently execute virtual staining of ovarian cancer pathological slices, and the quality of the generated virtual stained images is guaranteed. We have also compared with previous methods; the latter cannot exceed our proposed method in terms of image quality or evaluation accuracy. Our Code is available at https://github.com/menggerSherry/ImageStain.

## 2. Materials and Methods

### 2.1. Related Work

#### 2.1.1. Generative Adversarial Network

Generative Adversarial Network was first proposed by Goodfellow et al. [17]. Different kinds of GANs model have shown its remarkable data generation especially in the computer vision domain. Recently, successful research such as image generation [18–20], image-to-image translation [15, 21, 22], and superresolution [23, 24] shown remarkable result. Traditional structure of GAN contains two networks: a generator and a discriminator. The generator learns from a random noise to images which is same as the train set. The discriminator learns to distinguish the real image in the data set and the fake image generated by the generator. The propose of the idea of GAN can produce better image results through the continuous adversarial training between the generator and the discriminator. However, there are still some problems in GAN training, such as unstable training and model collapse.

#### 2.1.2. Conditional GANs

Traditional GAN model has shown very powerful data generation capabilities. However, we cannot artificially control the generation state of GAN and let the model generate the image we need. Mirza and Osindero [25] successfully solved this problem. Many researchers control GAN to generate data purposefully by imposing some conditions in training and introduce many conditional GAN models. Researchers have made many improvements to conditional GAN, making conditional GAN widely used. Research on the conditional GAN is widely welcomed in the face editing [26], domain transfer [27], and photo editing [28]. Today's conditional GAN has not only been widely used in the direction of computer vision but also began to receive attention in audio and language processing. As conditional GAN has been widely used, its problems have gradually emerged. During the training process, it is easy to fit only to several optimal directions, which eventually leads to the collapse of the model and loss of model diversity. At the same time, in the training process, user cannot control the training progress of the generator and the discriminator, making GAN very unstable during the training process.

#### 2.1.3. Improvement of GAN

Model collapse and training instability seriously affected the final experimental results. There are many aspects of research that have begun to solve these two fatal problems and have achieved good results. Raford et al. [20] use deep convolutional networks to design generators and discriminators and adopt batch normalization. The proposal of DCGAN solves the problem of unstable training and the model collapse. At the same time, applying CNN to the network structure can better adapt to the processing of images. Martin et al. [18, 19, 29] analyzed in detail the reasons for the collapse of the GAN model and the unstable training. They modified the loss of the original GAN to Wasserstein loss [18] and added a gradient penalty [19] so that the GAN model completely avoided these two problems.

#### 2.1.4. Image-to-Image Translation

The image-to-image translation has been a hot topic since GAN was proposed. Because of the wide range of uses of this type of problem, many researchers have begun research in this field. This issue was first raised by Isola et al. [21]. They modified the conditional GAN and finally achieved excellent image translation results. Today, image translation has achieved remarkable results in domain translation [15, 26], superresolution image synthesis [22, 30], video synthesis [31], etc. The problem we are facing now is the H&E staining of ovarian cancer pathological slices. Inspired by the above successful cases, we used the idea of conditional GAN to improve a new network structure and training strategy and finally realized this virtual staining of ovarian cancer. Through the final verification stage, we found that significant success has been achieved in both efficiency and effectiveness.

### 2.2. Construction of the Paired Data Set

Our goal is to finish the accurate staining of ovarian cancer tissue. This means that every cell structure can be accurately stained. Therefore, we intend to build a fully supervised image to image translation model. With reference to the method of Rivenson et al. [14], the unstained image is obtained by placing a fresh tissue section of ovarian cancer in a fluorescence microscope for direct observation. Then, performing elaborate staining on this fresh tissue to get the stained image. In this way, each unstained image corresponds to a stained image as a label. It is indeed feasible to construct a perfect data set by repeatedly conducting the above steps. The work of Rivenson et al. did give marvelous results. But when we implement their idea, we found that collecting so many fresh sections in a short time is indeed not an easy task, and it is laborious and tiring to do these jobs repeatedly. There is also a problem that the data set is limited. We have a large number of H&E staining images of ovarian cancer, but the number of autofluorescence images of fresh slices is very rare, which makes the distribution of the two sets of data very uneven. Due to some of the above problems, we decided to abandon the method of Rivenson et al. and propose a deep learning method to complete the construction of the above-paired data set under limited supervision conditions.

#### 2.2.1. CycleGAN Baseline

Unpaired image to image problem is an important problem. In many cases, building a paired data set takes a lot of time and work, but using unpaired image to image translation can avoid time-consuming data collection. The CycleGAN proposed by Zhu et al. [15] is a good model to solve such problems. Zhu et al. proposed a cycle consistency loss, ‖*F*_*X*⟶*Y*_ (*G*_*Y*⟶*X*_ (*x*)) − *x*‖_1,_ ‖*G*_*Y*⟶*X*_ (*F*_*X*⟶*Y*_ (*x*)) − *x*‖_1_ finished the translation of the domain *X* and the domain *Y*. Using this unsupervised method can effectively achieve conversion between two distributed data. But as mentioned above, the data distribution between our existing two domains is extremely uneven. In our experiment, we used the CycleGAN model to complete the data construction, but the results were very disappointing.

Figure 2(a) is the result of training using the CycleGAN model. We can see that there are a large number of sharp holes in the image. The input stained image's positions corresponding to these holes have normal textures, indicating that this model cannot effectively learn the features corresponding hole domain. We then introduce a large number of data augmentation methods based on the original CycleGAN, such as random jitter, random horizontal and vertical flips, random jitter rotation (first interpolate and zoom, then randomly rotate a small angle, and finally crop to the original image size), and elastic deformation [16]. We can observe the results as shown in Figure 2(b). The number of cavities is obviously reduced, and the overall image quality has been slightly improved, but the existence of cavities is still not completely resolved.

We zoomed on the position of the hole as shown in Figure 2(c). It can be found that the generator and discriminator in these positions did not play their role at all. We hypothesis that the feature distribution of the unstained image domain is sparser than the stained image domain's. The essence of domain to domain translation is to learn the features of images in a domain and then translate these features based on the supervision of the image feature rules of the target domain. Based on the above assumptions, when converting from a stained domain to an unstained domain, the features of the stained domain learned by the generator may be difficult to be reasonably represented by the limited positive sample image features of the unstained domain distribution. This will affect the discriminator's training on the area where these features are located. The generator synthesized a black hole in this area, which can make the discriminator think it is true, resulting in a train mode collapse in this area. With continuous training, the effect in areas with sufficient supervised positive sample features is getting better and better; this area remains unchanged, and the black hole continues to become obvious.

#### 2.2.2. Domain Consistency Network

When data augmentation is introduced, the number of samples theoretically increases, but with the increase in the number of data augmentation methods introduced, many augmented images may appear only a few times during training, which will cause the underfitting issue. We therefore introduce an input buffer to store the input image after a large amount of data augmentation and then randomly select the input image from the buffer as the input of the network. At the same time, in order to enhance the fitting ability of the network, we introduce the domain consistency loss. Specifically, a domain consistency discriminator is introduced to distinguish which domain the image belongs to. It participates in the training with the generator. In this way, through continuous training, the generator can synthesize images that are more accurate to a specific domain.

Figure 3 describes the structure of the domain consistency network and its training process. Where SepConv is the Deep Separable Convolution, LReLU is the LeakyReLU activation operation. The network first downsampling the input image on both sides three times to extract the effective features of the image, then fuses the two features and performs a series of convolution layers with 1 × 1 kernel to extract relevant information from the fused features and obtain a single-channel result. We ensure that the output dimension of the network is the same as the output dimension of the discriminator. In this way, real images with a large amount of data augmentation are first pushed into the buffer, and then, the buffer randomly selects two batches of images as the real image input of the domain consistency network. The domain consistency network learns that they belong to the same domain. The image generated by the generator and the real image randomly selected from the buffer are used as the input of the domain consistency network, and the network learns to distinguish that they belong to different domains. While learning to fool the discriminator, the generator also needs to fool the domain consistency network so that the domain consistency network thinks that the generated image and the real image are in the same domain.

We define the mapping *G*_1_ : *X*⟶*Y* as the conversion process from the stained image domain *X* to the unstained image domain *Y*, and its corresponding domain consistency network is *C*_1_. We can describe the domain consistency loss as:

(1) $$\begin{array}{c} L\left(G_{1},C_{1},X,Y_{1},Y_{2}\right)=E_{y∼p_{\text{data}}\left(y\right)}\left[{\left(C_{1}\left(\text{Aug}\left(Y_{1}\right),\text{Aug}\left(Y_{2}\right)\right)\right)}^{2}\right]+E_{x∼p_{\text{data}}\left(x\right)}\left[{\left(1-C_{1}\left(\text{Aug}\left(Y_{1}\right),G_{1}\left(X\right)\right)\right)}^{2}\right]. \end{array}$$

The Aug in Equation (1) represents the corresponding data augmentation; Aug(*Y*_1_) and Aug(*Y*_2_), respectively, represent the unstained image randomly selected from the input buffer after the augmentation transformation. Here, *G*_1_ tries to generate an unstained image *G*_1_(*x*) that is very close to the representative Aug(*Y*_1_) of the unstained image domain, and *C*_1_ tries to distinguish whether the two input images Aug(*Y*_1_) and Aug(*Y*_2_) are in the same domain. Like the idea of adversarial training, *G*_1_ tries to minimize the objective function of equation; *C*_1_ tries to maximize the objective function of Equation (1), which is expressed as min_*G*_1__max_*C*_1__*L*(*G*_1_, *C*_1_, *X*, *Y*_1_, *Y*_2_). Similarly, to ensure the balance of training, we use min_*G*_2__max_*C*_2__*L*(*G*_2_, *C*_2_, *Y*, *X*_1_, *X*_2_) to represent the domain consistency loss affecting the stained image.

The image shown in Figure 2(d) is the result of the unstained image synthesized by the generator after we introduce the domain consistency network. It can be found that compared with the results of the first two models, the result of Figure 2(d) is closer to the real image domain, the image quality has been significantly improved, and the sharp holes have become significantly smoother. Yet it is extremely frustrating that the issue of sharp holes has not been completely solved, and there are still unmatched black areas in the generated image.

#### 2.2.3. Modification of the Generator Network Structure

Let us revisit the reasons for the formation of sharp holes. A similar problem also occurred in the experiment of Karras et al. [32–34]. They observed that most images generated by StyleGAN [33] exhibit characteristic droplet-like artifacts that resemble water droplets. They think it is caused by the AdaIN problem in StyleGAN, and then, they canceled the normalization operation in StyleGAN2 [34], so that droplet-like artifacts can be effectively solved. The generator of the traditional CycleGAN model adopts the network structure proposed by Johnson et al. [35]. The design idea of the network is to perform deep feature fusion of the sampled feature maps by stacking residual blocks. And CycleGAN uses Instance Normalization after each convolution operation. Combined with the hypothesis of Karras et al., we believe that the key issue lies in Instance Normalization. Instance Normalization is to normalize each layer of feature maps separately, which may ignore the correlation between each layer of feature maps to a certain extent. Meanwhile, due to the structural particularity of the residual block, directly summing the residual and the result after convolution is likely to amplify the effect of Instance Normalization, thus creating this kind of hole.

We made a simple design on the basis of the original generator to completely solve this problem. Since Instance Normalization may affect the correlation between feature maps, we enhance the correlation of the network's feature channels. We first use the Xception block [36] instead of the original residual block. Xception block uses a depth-wise separable convolution, which is mainly composed of depth-wise convolution and point-wise convolution. The benefit of the depth-wise separable convolution is that the convolution's spatial correlation and the feature map channel correlation are operated separately, which reduces the number of training parameters and improves the influence of the convolution on the channel correlation. Next, in order to completely eliminate the problem of Instance Normalization, we replace the convolution operation in the upsampling process and downsampling with depth-wise separable convolution operation. Through the above modifications, we believe that the new generator can completely avoid the cavity problem.

Figure 2(e) is the inference result after training with the improved generator network. We can see that we have completely solved the hole problem, and the image quality was further enhanced. At the same time, through quantitative evaluation, we conclude that this method can construct a good unstained data set. We evaluated the quality of images generated by different methods, and the test results are shown in Table 1. From the evaluation results in the table, we can see that the quality of the images generated by our method far exceeds the state-of-the-art method. At the same time, we also submit the generated data to the doctor to judge, so that the doctor can distinguish the authenticity of the generated image. We have prepared 400 unstained images generated by different methods to allow doctors to judge the images within the specified time. According to the number of correct images, we can get the accuracy. The correct rate of each trial we recorded is shown in Table 2. It can be found that the accuracy of the images obtained by the previous methods is very low. Our analysis is due to the influence of the black holes in the generated images. When there are black holes in the generated image, the doctor will naturally distinguish the difference from the real image and consider the image to be a fake image. This may be why when we completely solve the hole problem, the accuracy of the image is doubled.

### 2.3. A Virtual Staining Method Specific to Tissue Texture

Through the above methods, we successfully constructed the paired data set composed of unstained images and stained images. We thus can regard virtual staining as an image-to-image translation problem. Today, many mature algorithms in the field of image-to-image translation have produced amazing results, yet whether these algorithms can be directly applied to this special domain remains to be verified. What we want is an image translation that is accurate to the tissue, so we need to build a more accurate image-to-image translation algorithm. In order to achieve this goal, we have made many modifications to the loss function, network structure, and training strategy.

#### 2.3.1. The Review of Image-to-Image Translation

Conventional image-to-image translation algorithms are usually based on the Pix2Pix baseline. Isola et al. [21] use UNet as the generator and use the patchGAN structure discriminator to discriminate images with accuracy to the patch. And the L1 loss is introduced on the basis of the conventional GAN loss to evaluate the pixel gap between the real image and the generated image. UNet was originally a dedicated network structure designed to handle cell structure segmentation tasks. It can effectively retain a lot of accurate and detailed feature information through layer-by-layer skip connections. At the same time, the patchGAN discriminator reduces the receptive field of the image to be determined, so that the discriminator has a stronger ability to distinguish the details of the image, which also promotes the quality of the generated image. We consider using the idea of Pix2Pix to perfect the model so that the model can better apply to the problems we are facing this time.

#### 2.3.2. A UNet Structure-Based Generator

The essence of the image translation task is that we input an image into the network; the network can learn various features of the image and then convert the original features of the image into the target features. We can simply regard the feature as the information that people can obtain by observing the image, specifically, the information that can perceive after the pixel value of the image is saw by the person. Therefore, the translation process from an image with original features to an image with another type of features can be conceded as the pixel value conversion of the image. From this perspective, image translation and semantic segmentation tasks are very similar, which is why the generator networks in the earliest image translation tasks (such as Pix2Pix [21]) are designed with the help of UNet networks. The UNet network was first used in the semantic segmentation task of the cell dimension. It uses skip connection to allow the network to effectively learn detailed features. Therefore, our task is also based on the UNet structure to design generator.

The process of using convolution to extract image feature values is a process of continuous dimensionality reduction of image feature data. In this process, the network must selectively learn to extract more representative features. On the contrary, some low-frequency, nonrepresentative features will be ignored in the feature extraction process. When we directly sample the dimensions of features, the network can only use these most representative features. In the process of directly decoding from high-frequency features to the target image, the network will ignore many low-frequency features, which makes the generated image quality very unsatisfactory. The introduction of skip connection is to fuse these low-frequency features with the features of the restoration process. This is why the image translation model using the UNet network as the generator can achieve great results.

So why do not we directly tell the network what characteristics we want to learn? We therefore deconstructed the original UNet network and designed a new generator. We call it the Parallel Feature Fusion Network (PFFN). Its network structure is shown in Figure 4. The stained image we input first enters the Average Pooling Sampling Block in Figure 4(a), and the network will perform the sampling work according to different sampling steps. Through the above operations, we obtain sampled images at different scales. Taking an input image with a size of 256 × 256 pixels as an example, after sampling with steps 6, 5, 4, 3, 2, and 1, respectively, the different scaled images with 8 × 8, 16 × 16, 32 × 32, 64 × 64, 128 × 128, and 256 × 256 are obtained. Through continuous downsampling operations, the image will lose many low-level aspects features but on the contrary can retain many high-level features. For example, after we sample a cell tissue image, we can see that the high-level aspect features of the image such as the shape of the cell, but we cannot see the low-level features that are lost after sampling, such as the detailed structure within the cell.

After receiving the input images of six scales, we input the images of each scale into the corresponding Parallel Feature Extraction Block in Figure 4(b). Each feature extraction network is designed based on the UNet structure, and the detailed network implementation is shown in Figure 5. The function of the FromRGB module in Figure 5(a) is to convert the image into a feature map of 512-dimensional channels. In the entire network, we stipulate that the feature map is 512 dimensions. We design three branches in FromRGB module, and each branch adopts different sampling methods. Finally, the feature maps of different sensory scales sampled by different sampling methods are deeply fused and used as the input of the improved UNet network in Figure 5(b).

Due to the different sampling scales of input images of different scales, we design three UNet structures as the feature extraction network, named UNet_2_, UNet_4_, and UNet_6_, respectively. The subscripts indicate the feature sampling depth of the UNet. The network structure shown in Figure 5 is UNet_2_. What differs from the traditional UNet is that we added the additional skip connections. Unlike the conventional UNet network, we have introduced additional skip connections from the upper layer to the lower layer on the UNet. As we mentioned, every time the network passes through a convolutional layer, some low-frequency features are lost. The original UNet skip connection only guarantees the low-frequency feature transfer to the same layer, but the lower layer may also need the low-frequency feature of the upper layer. We therefore introduced a skip connection from the upper layer to the lower layer so that the bottom layer can also learn effective low-frequency features. This design is very similar to the idea of UNet3+ [37], but we removed the skip connection to the deeper layer. First of all, the number of layers of our three UNet networks is not deep enough. The introduction of so many skip connections may not be significantly improved. On the contrary, it will bring a greater amount of calculation. This new structure diagram of UNet is shown in Figures 5 and 6 where the red arrows indicate the new skip connection we added. We used Unet_6_ and UNet as the generator to train the models separately and evaluate the quality of the generated images. It can be seen from Table 3 that the image quality generated by UNet_6_ is improved compared with the traditional UNet, where the FID decreased by about 2-3 and the Inception Score decreased by about 0.01-0.04. However, the network depth of UNet_6_ is only 6 layers, and the depth of UNet reaches 8 layers. It can be proved that UNet_6_ has a powerful feature learning ability within a limited sampling field.

We specify that 8 × 8 and 16 × 16 input images use UNet_2_ network, 32 × 32 and 64 × 64 input images use UNet_4_ network, and 128 × 128 and 256 × 256 input images use UNet_6_ network. In the process of continuous sampling of images with 256 × 256 pixels to 8 × 8, the lower resolution image retains the higher-level aspect features, which can be learned by using the shallow network structure like UNet_2_. As the image pixels increase, the UNet network structure continues to deepen, and the effect of UNet will continue to be highlighted. The low-level aspect features of high-resolution images can be learned through the deeper network like UNet_4_ and UNet_6_. In this way, the network can learn the image features of each level of the sampling module according to our wishes, and the resulting feature maps cover the feature values of the image from coarse to fine. We finally introduce an upsample process to continuously fuse these features to obtain the final output image. In the process of upsample, we also introduce skip connection to ensure the feature of high-level aspects to propagate down better. Compared with the traditional UNet network as the generator, the network designed by us has a wider reception field, and the image obtained has a stronger performance ability, while covering all the characteristics of UNet. From Table 3, compared with the image quality generated by UNet, the FID of the image generated by using our PFFN network as a generator was reduced by about 3-9, and the Inception Score was reduced by about 0.1-0.2. Compared with the image FID generated by UNet_6_, the FID was reduced by about 1-8, and the Inception Score was reduced by about 0.1-0.2.

#### 2.3.3. Choice of Loss Function

The most commonly used loss functions of traditional GANs are cross-entropy loss and *L*_2_ loss. These loss functions have proven their feasibility in GAN training through a large number of experiments. But there are also many studies show that using these two loss function optimization models in GAN's training will cause very terrible results. Moreover, many drawbacks of GAN, such as mode collapse and training instability, are caused by the use of these instable loss functions. We used this kind of loss function to train in the experiment, yet the result is not what we expected. Therefore, choosing an appropriate loss function is very important in this experiment.

In this experiment, we consider using two robust loss functions: Wasserstein loss with gradient penalty [18, 19] and Logistic loss [33] with R1 regularization [38, 39] as the training loss function. Wasserstein distance is simple and direct compared to the original loss function and highly correlates with the quality of the synthesized image of the generator. Using Wasserstein loss may be a good choice. Logistic loss is applied in the StyleGAN paper by Karras et al. [33]. He used this loss as the adversarial loss and generated the high-resolution face images. Both of these two loss functions have very good performance. In order to verify which loss function can be better applied to our virtual staining experiment, we use these functions to train the model and evaluate the generator by the quality of the image. As shown the results in Table 3, we find that the image quality synthesized by the generator trained with the Wasserstein loss (Equation (2)) is better.

(2) $$\begin{array}{c} L_{\text{gan}}\left(G,D,x,y\right)=E_{x∼p_{\text{data}}\left(x\right)}\left[D\left(x,G\left(x\right)\right)\right]-E_{y∼p_{\text{data}}\left(y\right),x∼p_{\text{data}}\left(x\right)}\left[D\left(x,y\right)\right]-\lambda_{gp}E_{\hat{x}∼p_{\text{data}}\left(\hat{x}\right)}\left[{\left\|\left(\nabla_{\hat{x}}\right.D\left(\hat{x}\right)\right\|}_{l2}^{2}-{\left.1\right)}^{2}\right]. \end{array}$$

The traditional image translation model usually introduce an additional L1 loss (Equation (3)) based on adversarial loss; its function is to narrow the global gap between the real image and the generated image. But the introduction of this loss will make the image blurred and attenuate the quality of the generated image. To get a higher quality image, we need a sturdy loss function to act on the generator. Wang et al. [22] used the feature matching loss (Equation (4)) in the high-resolution image translation task of the Cityscapes data set and got flawless results. We introduced this loss into the training of the generator and found that the effect has been significantly improved through the final evaluation results. According to the results of our experiment, we choose Wasserstein loss in the adversarial loss, as shown in the Equation (2), where ${𝔼}_{\hat{x}∼p_{\text{data}}\left(\hat{x}\right)}\left[{\left\|\left(\nabla_{\hat{x}}\right.D\left(\hat{x}\right)\right\|}_{l2}^{2}-{\left.1\right)}^{2}\right]$ represents the gradient penalty for the $\hat{x}$, which is the random interpolating of the positive sample and the generated sample. In order to reduce the global difference between the generated image and the real image, we retain the L1 loss as shown in Equation (3). In order to further improve the quality of the generated image, we increase the feature matching loss, as shown in the Equation (4), where *N* represents the number of layers of the discriminator.

(3) $$\begin{array}{c} L_{\text{pix}}\left(G,x,y\right)=E_{x∼p_{\text{data}}\left(x\right),y∼p_{\text{data}}\left(y\right)}\left[{\left\|y-G\left(x\right)\right\|}_{l1}\right], \end{array}$$

(4) $$\begin{array}{c} \begin{array}{r} L_{\text{fm}}\left(G,D,x,y\right)=E_{x∼p_{\text{data}}\left(x\right),y∼p_{\text{data}}\left(y\right)}\left[\frac{1}{N}\overset{N}{\underset{i=1}{\sum }}\left({\left\|D\left(x,y\right)-D\left(x,G\left(x\right)\right)\right\|}_{l1}\right)\right]. \end{array} \end{array}$$

The model loss we finally get is expressed by the following Equation (5). We use the gradient descent method to solve the following equation: *G*_opt_, *D*_opt_ = argmin_*G*_max_*D*_*L*(*G*, *D*, *x*, *y*). Finally, we can get the optimal solution of the staining model.

(5) $$\begin{array}{c} \begin{array}{c} L\left(G,D,x,y\right)=L_{\text{gan}}\left(G,D,x,y\right)+\lambda_{\text{pix}}L_{\text{pix}}\left(G,x,y\right)+\lambda_{\text{fm}}L_{\text{fm}}\left(G,D,x,y\right). \end{array} \end{array}$$

## 3. Results and Discussion

Through the above training, we have successfully generated H&E staining of ovarian cancer pathological slices.  Figure 7 is the result comparison between the generated virtual stained image and the real H&E staining image. Intuitively, the gap between the real and the fake is quite hard to distinguish, but for this method to be better used in medical products, we need to compose a series of evaluations on these virtual stained images we generate.

### 3.1. Artificial Pathology Analysis

A successful virtual staining section can express the correct pathological characteristics; otherwise, it will seriously affect the doctor's pathological diagnosis. To evaluate the generated pathological slices more subjectively, we invited three professional doctors to analyze the difference between the image generated by our model and the real image and evaluate whether the staining for these images is successful. After evaluating each image, we can roughly get the staining accuracy of our model. Since it is a heavy task to evaluate a large number of images, we only randomly selected 200 images as the evaluation data, and the final results obtained are shown in Table 4. According to the doctor's evaluation results in Table 4, the staining accuracy of our method reaches 97%, which proves that our method has achieved a perfect staining effect. However, our verification case is only 200 cases, which cannot well represent the overall effect. We need to add evaluation cases in the next period of treatment.

### 3.2. Visual Simulation Analysis

It was mentioned in the previous section that direct subjective analysis by doctors can certainly get a good score result, but it will consume a lot of time and work, and the results of the evaluation using a small number of samples do not have a good overall representativeness. In particular, our model can generate a large number of H&E staining models in a short time, which is very unrealistic for doctors to perform analysis and evaluation.

To overcome this problem, we propose a method based on deep learning to simulate the visual analysis of doctors. The H&E staining sections of real ovarian cancer we selected have detailed pathological analysis results, and each section doctor clearly marked a cancer lesion and tumor type. We can train a classification network based on the data set composed of real images based on the above annotations. We can think that the trained classification network has the doctor's focus classification ability. Since the generated pathological stained slices should have the same pathological characteristics as the corresponding real stained slices, we use the pretrained classification network to make inference and prediction tumor type results for the corresponding generated virtual stained images. Finally, we calculate the difference between the result of the generated image and the real result to get the final accuracy. This accuracy can approximately represent the quality of the lesion features based on the image generated by our model.

First of all, each stained image in our data set is annotated by professional doctors according to the four types of tumors. Next, we use these labeled data sets to train a VGG16 classification network. The classification accuracy of the trained network reached about 97%. We can think that this VGG network has a strong ability to distinguish ovarian cancer tumor types. Then, we use the trained VGG network to predict the stained ovarian cancer sections we generated and calculate the accuracy. If the prediction of the generated image is correct, it can indicate that the virtual stained slice we synthesized expresses the correct feature of the lesion. We think it is reasonable to apply such images to pathological analysis. Finally, the accuracy of the proposed method reached 95%. We can conclude the final difference of virtual staining to be 2%. It can be proved that our method has reached the standard of pathological analysis of ovarian cancer.

## 4. Conclusions

We provide a more efficient solution for H&E staining of ovarian cancer pathological sections. Using our method can be very effective to save time and quickly assist the doctor in diagnosis. We have used many evaluation methods. From the results, the quality of the stained image generated by our method is very perfect. At the same time, we have also proposed an effective autofluorescence image generation algorithm in the absence of valid data, which can save time-consuming and laborious data preparation time in many cases. In the next research, we will carry out research on virtual staining of more pathological tissues in order to realize a more extensive virtual staining technology.

## Figures and Tables

**Figure 1:** Overview of this virtual staining process: (a) the overview of this domain translation method; (b) overview of the virtual staining process.

**Figure 2:** Comparison of the results of using different trained models to construct data sets: (a) results generated by CycleGAN model; (b) results synthesized by the improved CycleGAN model; (c) enlarge some cavity area of the synthesized image; (d) results after introducing domain consistency network training; (e) result of using our modified generator structure and domain consistency network.

**Figure 3:** Training the domain consistency network.

**Figure 4:** The structure of Parallel Feature Fusion Network.

**Figure 5:** Network structure of feature extraction module (UNet_2_). (a) FromRGB module. This module extends low-dimensional images to higher dimensional feature maps. (b) Feature extraction module based on UNet_2_.

**Figure 6:** The UNet structure introducing additional skip connections.

**Figure 7:** Virtual staining result display on pathological sections of ovarian cancer.

**Table 1:** Comparison of the quality of unstained images using different methods.

	CycleGAN	Improved CycleGAN	Ours	Ours (with separable Conv)
IS ↓	1.590	1.700	1.407	1.311
FID ↓	471.421	360.029	235.410	175.969
MS ↓	0.883	0.873	0.794	0.717

**Table 2:** Accuracy results of unstained images synthesized using different methods.

	CycleGAN	Improved CycleGAN	Ours	Ours (with separable Conv)
Doctor 1	12.50%	1.25%	24.25%	77.5%
Doctor 2	3.50%	5.50%	39.5%	86.5%
Doctor 3	0.00%	1.50%	55.50%	93.50%

**Table 3:** Comparison of image quality using different loss functions and generator network structures.

Network	Loss function	FID ↓	IS ↓
UNet	*L*_*l*_2__	57.6092	1.3405
	*L*_wgan_	54.1733	1.4687
	*L*_logistic_	56.1733	1.4687
	*L*_*l*_2__ + *L*_fm_	59.4684	1.4720
	*L*_wgan_ + *L*_fm_	58.1196	1.4720
	*L*_logistic_ + *L*_fm_	56.1639	1.4432

UNet_6_	*L*_*l*_2__	54.1436	1.3928
	*L*_wgan_	50.8299	1.4256
	*L*_logistic_	52.4708	1.3865
	*L*_*l*_2__ + *L*_fm_	51.3790	1.3907
	*L*_wgan_ + *L*_fm_	55.2754	1.4852
	*L*_logistic_ + *L*_fm_	49.3387	1.4073

PFFN (ours)	*L*_*l*_2__	54.8384	1.3835
	*L*_wgan_	49.1167	1.3903
	*L*_logistic_	49.6818	1.4124
	*L*_*l*_2__ + *L*_fm_	49.3575	1.3238
	*L*_wgan_ + *L*_fm_	47.0977	1.3505
	*L*_logistic_ + *L*_fm_	48.8730	1.2158

**Table 4:** Staining accuracy of our model analyzed by three doctors.

	Doctor 1	Doctor 2	Doctor 3
Samples with successful staining	190	196	194
Accuracy	95%	98%	97%

## Data Availability

The data we use is mainly composed of the TCGA ovarian cancer database and the clinical data. TCGA ovarian cancer data can be obtained from https://portal.gdc.cancer.gov/. Considering the privacy of patients, we cannot open access to our clinical data.
